# The Clinical Efficacy of *Ginkgo biloba* Leaf Preparation on Ischemic Stroke: A Systematic Review and Meta-Analysis

**DOI:** 10.1155/2021/4265219

**Published:** 2021-12-09

**Authors:** Shuang Zhao, Hong Zheng, Yawei Du, Runlei Zhang, Peilin Chen, Rong Ren, Shengxian Wu

**Affiliations:** ^1^Dongzhimen Hospital, Beijing University of Chinese Medicine, No. 5, Haiyuncang, Dongcheng District, Beijing 100700, China; ^2^First Clinical Medical School, Beijing University of Chinese Medicine, No. 11, Bei San Huan Dong Lu, Chaoyang District, Beijing 100029, China

## Abstract

**Background:**

*Ginkgo biloba* leaf preparations (GLPs) are widely used in ischemic stroke, and uncertainty remains regarding their clinical efficacy. To evaluate systematically the clinical efficacy and safety of GLPs in the treatment of ischemic stroke, we examine evidence from randomized controlled trials (RCTs).

**Methods:**

We examine studies published prior to November 2021 that were found from searching the following sources: PubMed, China National Knowledge Infrastructure (CNKI), WANFANG DATA, Chongqing VIP (CQVIP) databases, and Chinese Biomedical Literature (CBM). We evaluated the quality of the included references according to the Cochrane Manual of Systematic Evaluation and Meta-analysis (MA) performed using RevMan 5.2 software.

**Results:**

We included a total of 13 RCTs with clinical therapeutic effects, the National Institute of Health Stroke Scale (NIHSS), Barthel Index (BI), hemorheology index, and adverse reaction index as evaluation criteria. There were 631 cases in the observation group and 629 cases in the control group. MA results showed the following: NIHSS WMD = −3.89, 95% CI: [−4.22, −3.56], *I*^2^ = 19%, *P* < 0.00001. This index is often used with nerve injury and can also be used to judge the recovery of nerve function. A lower score means less nerve damage and a better chance of recovery. The BI results were WMD = 11.30, 95% CI: [9.83, 12.77], *I*^2^ = 7%, *P* < 0.00001. This index was used to assess patients' ability to take care of themselves, with a higher score indicating a stronger ability to live independently. Clinical effective rate results were WMD = 3.79, 95% CI: [2.49, 5.78], *I*^2^ = 0%, *P* < 0.00001, and this measure can be used to evaluate the effect of treatment clearly and objectively. Hemorheological index results show that plasma viscosity has WMD = −0.16, 95% CI: [−0.20, −0.12], *I*^2^ = 40%, *P* < 0.00001 and fibrinogen (FIB) has WMD = −1.13, 95% CI: [−1.23, −1.04], *I*^2^ = 0%, *P* < 0.00001. Plasma viscosity is mainly related to the amount of fibrinogen, and fibrinogen degradation is an important function of the fibrinolytic system. The imbalance of the fibrinolytic system plays an important role in the pathogenesis of cerebral infarction. Fibrinogen is a risk factor of ischemic cerebrovascular disease. Studies have shown that the infarct size of patients with secondary cerebral infarction after CEREBRAL infarction is correlated with their FIB level. In addition, FIB elevation is also one of the risk factors for early infarction after thrombolysis. Therefore, FIB can be used as a detection index for the prevention of cerebral infarction recurrence adverse reactions. Our MA results for FIB show WMD = 0.81, 95% CI: [0.38, 1.73], *I*^2^ = 0%, *P* = 0.58, and RR < 1.

**Conclusion:**

The existing clinical evidence shows that GLP has a good therapeutic effect on patients with ischemic stroke and can improve their hemorheology indices. In addition, GLP is shown to be relatively safe.

## 1. Introduction

Cerebrovascular disease is one of the leading causes of death in China, where it is estimated that there are 13 million stroke patients [1]. Among the existing types of cerebrovascular diseases in China, about 70% of the patients suffer from ischemic stroke [2]. Ischemic stroke is characterized by a high mortality rate, a high teratogenicity rate, and a high recurrence rate. It not only seriously affects the quality of life of patients but can also cause a serious economic burden on those afflicted and their families [3].

In recent years, a number of studies have provided evidence that *Ginkgo biloba* leaf extract has natural antioxidant properties, can specifically scavenge a variety of oxygen free radicals, can help activate antagonistic platelet activation factor and other biological activities, can significantly expand the cerebrovascular system, and can improve the symptoms of cerebral hypoxia [4–6]. The active ingredient in *Ginkgo biloba* ginkgolide has been shown to have a variety of neuroprotective and reparative effects that can help maintain the blood-brain barrier; reduce brain edema; improve energy metabolism; help with antioxidation, anti-inflammation, and antiapoptosis; promote angiogenesis; and provide a therapeutic effect for ischemic stroke [7].

However, the clinical use of *Ginkgo biloba* is not just limited to the basic leaves. Leaf preparations can also include ginkgo ketone ester dripping pills, ginkgo ketone ester dispersing tablets, Shuxuening injections, ginkgo diterpene lactone glutamine injections, ginkgo lactone injections, and ginkgo damo. With the wider application of GLPs across the globe, reports of adverse events have been gradually increasing as well; the most common adverse events are allergic reactions and abnormal bleeding [8, 9].

Ginkgo acid, in particular, which is a toxic substance in *Ginkgo biloba* leaves, has been shown to be a major cause of such allergies [10]. In addition, the ginkgo substance ginkgolide is a natural platelet antagonist with antiplatelet effects [11], and this may increase bleeding when used in combination with anticoagulants. It is not yet clear whether the adverse reactions of *Ginkgo biloba* preparations are individual or common.

In this paper, we searched RCTs of GLP in the treatment of ischemic stroke that were published since the establishment of each of our databases in order to evaluate the clinical efficacy and safety of GLP in the treatment of ischemic stroke and to provide a reference for the clinical treatment of ischemic stroke.

## 2. Methods and Materials

We performed our MA according to the Cochrane Handbook for Systematic Reviews of Interventions [12] and presented our results based on Preferred Reporting Items for Systematic Reviews and Meta-Analyses guidelines [13].

### 2.1. Literature Search

Two researchers (Shuang Zhao and Run-lei Zhang) searched PubMed, CNKI, WANFANG DATA, CQVIP, and CBM databases from their respective inception dates to November 2021. The search terms used were (in pseudo-logic): (stroke OR cerebral infarction OR ischemic stroke) AND (ginkgo OR Ginkgo biloba OR ginkgo biloba leaf preparation) AND (randomized controlled trial).

### 2.2. Inclusion and Exclusion Criteria

We abided by the participants, interventions, comparisons, outcomes and study design (PICOS) approach in establishing our inclusion criteria, which were as follows: (1) patients must have met the accepted diagnostic criteria for stroke with no restrictions on gender, age, BMI, or other measures. (2) We compared GLP with other interventions, and the possible comparisons were GLP plus conventional treatments versus conventional treatments. (3) We only included studies that reported at least one of the following outcomes: NIHSS, clinical therapeutic effect, BI, adverse reactions, plasma viscosity level, or fibrinogen.

The exclusion criteria were as follows: (1) review, experience, case reports, case reports, conference reports, animal experiments, and other literature; (2) duplicate publications, duplicate data, or incomplete literature; (3) intervention measures for other traditional Chinese medicine, Chinese patent medicine, acupuncture and massage, and other traditional Chinese medicine treatment literature; and (4) the observation group or control group had fewer than 20 cases or the total number was less than 40 cases.

No language restriction was applied.

### 2.3. Study Selection

Our reviewers worked in pairs. They first identified the articles that met the inclusion criteria through the title and abstract and then independently verified this through the full text.

### 2.4. Data Collection Process

Two researchers (Pei-lin Chen and Rong Ren) independently extracted the following information using predesigned forms: lead author, publication year, details of intervention measurement, sample size, ages of the participants, outcomes, and adverse events. In cases of disagreement between two reviewers from a pair, a third author or group discussion decided on inclusion or exclusion.

### 2.5. Risk of Bias Assessment

The methodological quality of the included studies was assessed by two researchers (Ya-wei Du and Sheng-xian Wu) according to the Cochrane handbook 5.1.0 [12]. Bias risk assessment was conducted from 7 items: random sequence generation, allocation concealment, blinding of researchers and subjects, blinded evaluation of study outcomes, integrity of outcome data, selective reporting of study results, and other biases. Green, yellow, and red colors with “+,” “−,” and “?” symbols denote “low risk bias,” “high risk bias,” and “unclear,” respectively, and the included literature was evaluated one by one. Disagreements were resolved through discussion with a third researcher (Hong Zheng).

### 2.6. Statistical Analysis

We used RevMan 5.2 software to process and analyze our extracted data. Dichotomous data were analyzed using risk ratios (RRs) and continuous variables using mean differences (MDs) with 95% confidence intervals (CIs). The *I*^2^ statistic was used to evaluate the heterogeneity among studies. If *I*^2^ < 50% and *P* ≥ 0.1, then heterogeneity was small, and we chose the fixed-effect model for analysis. If *I*^2^> is 50% or *P* ≤ 0.1, then heterogeneity was large, and we chose the random-effects model to analyze the causes of heterogeneity. Subgroup analysis or sensitivity analysis was performed if necessary. We also elect that a *P*statistic less than 0.05 indicates statistically significant results. When more than 10 articles were included in an outcome index, funnel plots were used to determine whether there was publication bias.

## 3. Results

### 3.1. Literature Selection

A total of 630 published articles were retrieved, including 210 from WANFANG DATA, 198 from CNKI, 200 from CQVIP, and 22 from Pubmed, imported into NoteExpress literature management software, and then removed 350 duplicate references. We also excluded 70 articles, including academic papers, nonclinical randomized controlled trials, academic conferences, reviews, empirical medical cases, and knowledge lectures. In addition, we eliminated 120 irrelevant and unusable articles on interventions after reading the article titles and abstracts. After excluding studies with fewer than 20 participants in the control or treatment group, or 40 total participants, and excluding 77 articles that had the same author and the same type of research, 13 RCTs remained to be included in our MA. The screening process is shown in Figure 1.

### 3.2. Characteristics of the Included Studies

A total of 13 articles meeting our criteria were included in the study, totaling 631 cases in the observation groups and 629 cases in the control groups. The included evaluation indices were clinical therapeutic effect in 9 articles, NIHSS in 7 articles, BI score in 5 articles, plasma viscosity level comparison in 6 articles, fibrinogen comparison in 4 articles, and the occurrence of adverse reactions in 5 articles (see Table 1).

### 3.3. Risk of Bias Assessment

All 13 articles randomly assigned patients to the observation group or the control group. Specifically, of the 8 articles that used the random number method (low risk of bias), two articles did not mention the specific random method (unclear risk), and 3 of them may have adopted an inappropriate random method (high risk). None of the 13 studies described allocation concealment, double-blindness among participants, or blinding of outcome assessment (unclear risk).

All studies had dropout rates of less than 20%, so they were all rated as low risk in terms of incomplete outcome data. Seven studies failed to report adverse events. The risk assessments of the 13 references are shown in Figure 2.

### 3.4. NIHSS

A total of 7 articles [14, 15, 19, 20, 22, 24, 26] used NIHSS as an evaluation index. Due to the presence of clinical heterogeneity in the index, we adopted a random-effects model for combined analysis, and the total combined results are as follows: WMD = −3.89, 95% CI: [−4.22, −3.56], *I*^2^ = 19%, and *P* < 0.00001. The difference of NIHSS between the observation groups and the control groups is statistically significant, and the heterogeneity was small. This indicates that the use of GLP may better improve the NIHSS, as shown in Figure 3.

### 3.5. Clinical Therapeutic Effect Evaluation

A total of 9 articles [14, 15, 19, 20, 22–26] used the clinical therapeutic effect as an evaluation index. Again, due to the presence of clinical heterogeneity in this index, we adopted a random-effects model for combined analysis, and the total combined results are as follows: WMD = 3.79, 95% CI: [2.49, 5.78], *I*^2^ = 0%, and *P* < 0.00001. The difference of clinical therapeutic effect between the observation group and the control group was statistically significant, and the heterogeneity was small. This suggests that the combined use of GLP can achieve better clinical efficacy, as shown in Figure 4.

### 3.6. Barthel Index

A total of 5 articles [15, 23–26] used BI as an evaluation index. Once again, due to the presence of clinical heterogeneity in this index, we adopted a random-effects model for combined analysis, and the total combined results are as follows: WMD = 11.30, 95% CI: [9.83, 12.77], *I*^2^ = 7%, and *P* < 0.00001. The difference of BI between the observation group and the control group was statistically significant, and the heterogeneity was small, again indicating that the use of GLP can improve the BI and improve living ability, as shown in Figure 5.

### 3.7. Plasma Viscosity Comparison

A total of 6 articles [16, 19, 21, 25] used plasma viscosity comparison as an evaluation index. Again, due to the presence of clinical heterogeneity in this index, we adopted a random-effects model for combined analysis, and the total combined results are as follows: WMD = −0.16, 95% CI: [−0.20, −0.12], *I*^2^ = 40%, and *P* < 0.00001. The difference of plasma viscosity between the observation group and the control group was statistically significant, and the heterogeneity was small. This too indicates that the use of GLP can improve plasma viscosity, as shown in Figure 6.

### 3.8. Fibrinogen Comparison

A total of 4 articles [16, 19, 21, 26] used fibrinogen comparison as an evaluation index, and again, due to the presence of clinical heterogeneity in this index, we adopted a random-effects model for combined analysis, and the total combined results are as follows: WMD = −1.13, 95% CI: [−1.23, −1.04], *I*^2^ = 0%, and *P* < 0.00001. The difference of fibrinogen between the observation group and the control group was statistically significant, and the heterogeneity was small, once again indicating that the use of GLP can reduce the level of fibrinogen, as shown in Figure 7.

### 3.9. Adverse Reactions Comparison

A total of 5 articles [17, 18, 23, 24, 26] used the comparison of adverse reactions as an evaluation index. Again, due to the presence of clinical heterogeneity in this index, we adopted a random-effects model for combined analysis, and the total combined results are as follows: WMD = 0.81, 95% CI: [0.38, 1.73], *I*^2^ = 0%, and *P* = 0.58, *RR* < 1. The difference of adverse reactions between the observation group and the control group was statistically significant, and the heterogeneity was small. This indicates that the number of ADR in the observation group is less than that in the control group, suggesting that the combined use of GLP and other interventions did not increase, at least at the same time, and may even have reduced the occurrence of ADR, as shown in Figure 8.

## 4. Discussion

The treatment of ischemic stroke can have different effects according to different times of intervention. Studies [27, 28] have shown that treatment in the early stage of stroke is of great significance to the recovery effect and the prevention of the recurrence of stroke. Zhu et al. [29] studied the effect of intensive medical treatment on acute ischemic stroke. They found that, in addition to controlling blood pressure, blood lipid, blood glucose, and other indicators and guiding patients to improve their poor lifestyle, an intensive medical treatment plan was studied. Their drug treatment scheme was as follows: Patients first received a dose of aspirin of 100∼300 mg/d, atorvastatin calcium 60∼80 mg/d, and clopidogrel 300 mg/d. After that, the dosage of aspirin was reduced to 100 mg/d, atorvastatin calcium remained at 60∼80 mg/d, and clopidogrel was adjusted to 75 mg/d, which continued for 90 days. Their findings suggest that intensive medical treatment during the acute phase of stroke can promote the recovery of neurological function in patients but does not increase the risk of adverse outcomes. Aspirin is now recognized as an effective means to prevent recurrent stroke [30]. However, other clinical studies report that, for patients with aspirin resistance [31, 32], clopidogrel is usually used instead of or in combination with aspirin. Other clinical studies also show that sometimes combined use is not effective. In addition, a higher dose of aspirin can increase the risk of bleeding, and clopidogrel is not widely accepted due to its high price. Studies [33, 34] have shown that aspirin combined with GLP can reduce aspirin resistance under a regime of low-dose aspirin and can help to avoid adverse reactions from high-dose aspirin at the same time. Moreover, GLP has a high cost-potency ratio. Therefore, while aspirin is the preferred drug for the secondary prevention of stroke, GLP can be used as a complementary therapy.

*Ginkgo biloba* is a deciduous perennial tree of the genus *Ginkgo* and the family *Ginkgoaceae*. Although once far more widespread than today, its leaves, kernels, and outer seed skins contain medicinal ingredients, and it is referred to in China as the “living fossil with treasure all over the body.” Ginkgo has been used as medicine for more than 600 years, and its efficacy was first recorded in “Shennong Ben Cao Jing.” Historically, China realized the medicinal value of ginkgo very early on. Li Shizhen in the Ming Dynasty wrote in his Compendium of Materia Medica that “Ginkgo enters the lung meridian, improves lung qi, eases asthma and reduces bowel movements.”

Modern research on ginkgo began in the 1950s. German scientist Dr. Willmar Schwabe found an optimal composition ratio in *Ginkgo biloba* extract (GBE) to maximize the medicinal value of *Ginkgo biloba* leaves. The resulting standard product is called EGb761. Chinese medicine practitioners believe that *Ginkgo biloba* leaves have the effect of activating blood and nourishing the heart, astringing the lungs, and restraining the intestine [35]. The seed kernels have been found to moisten the lungs, relieve asthma, relieve cough, diuresis, stop white turbidity, kill insects, and reduce the symptoms of hangover, among other effects.

According to current studies, the main active ingredients of *Ginkgo biloba* leaves are ginkgo flavonoids and *Ginkgo biloba* terpene lactone, both of which can improve blood flow and inhibit platelet aggregation [36]. A large number of experiments have also shown that *Ginkgo biloba* leaf extract can scavenge free radicals, protect neuronal cell membranes, and inhibit cell apoptosis induced by free radicals [37]. *Ginkgo biloba* leaf is widely used in the treatment of the cardiovascular system, nervous system, respiratory system and other fields and has become renowned for its curative effects. It has a good effect on the treatment of ischemic stroke, subarachnoid hemorrhage, senile dementia, vascular dementia, ischemic heart disease, hyperlipidemia, asthma, chronic pulmonary heart disease, sudden deafness, diabetic peripheral neuropathy, cancer, and many other diseases [38].

However, with the wider application of GLP in clinical practice, there have been more and more reports on the occurrence of adverse reactions, and there is a lack of evidence-based medicine to evaluate GLP's efficacy and safety. MA provides a comprehensive and complete reference for the use of clinical GLP. This paper systematically analyzed the experimental data of 13 included GLPs in the treatment of ischemic stroke. Our MA results show that NIHSS results were as follows: WMD = −3.89, 95% CI: [−4.22, −3.56], *I*^2^ = 19%, and *P* < 0.00001; BI results were as follows: WMD = 11.30, 95% CI: [9.83, 12.77], *I*^2^ = 7%, and *P* < 0.00001; clinical effective rate results were as follows: WMD = 3.79, 95% CI: [2.49, 5.78], *I*^*2*^ = 0%, and *P* < 0.00001; plasma viscosity results were as follows: WMD = −0.16, 95% CI: [−0.20, −0.12], *I*^2^ = 40%, and *P* < 0.00001; fibrinogen results were as follows: WMD = −1.13, 95% CI: [−1.23, −1.04], *I*^2^ = 0%, and *P* < 0.00001; and adverse reaction results were as follows: WMD = 0.81, 95% CI: [0.38, 1.73], *I*^2^ = 0%, and *P* = 0.58, *RR* < 1.

In all cases, we found that the combined effect size was statistically significant. In this study, clinical therapeutic effect, NIHSS, and BI were used as the main indicators. According to the results of our MA, GLP has a positive effect on the treatment of ischemic stroke, and it has a significant improvement effect on the neurological function and the ability to carry on daily living for patients with ischemic stroke. Using hemorheological indices (plasma viscosity and fibrinogen) as secondary measures, our MA suggests that GLP can change hemorheological indices related to ischemic stroke. Some studies have shown that fibrinogen is an important factor that affects the occurrence of stroke, and researchers speculate that increased fibrinogen content is a predictor for the occurrence of ischemic stroke [39]. Other studies have shown that fibrinogen can promote platelet aggregation [40]. Therefore, we speculate that GLP can aid ischemic stroke patients by improving plasma viscosity and reducing the level of fibrinogen.

However, considering that the test results of hemorheology indices are not necessarily positively correlated with clinical symptoms and conditions, such test results can only provide a reference for clinical treatment.

In the included literature, there were 14 adverse events in the observation groups and 17 in the control groups. The proportion of the number of adverse events in the observation group and the control group was similar, and most of the adverse symptoms disappeared after the end of treatment without the need for special treatment, indicating that the use of GLP did not cause serious adverse reactions. Ginkgo acid is one of the main toxic components in *Ginkgo biloba*. At present, the methods of *Ginkgo biloba* deacidification include microwave-assisted extraction, organic solvent extraction, resin extraction, ultrasound-assisted extraction, and supercritical carbon dioxide extraction [41].

Based on clinical safety considerations, the content of ginkgo phenolic acid has become an important control index in the quality standard of ginkgo drug semifinished products as well [42]. With the growing use of *Ginkgo biloba*, we may expect that its technology will continue to progress, and its quality control standards may become more and more strict. In addition, according to current studies, the occurrence of bleeding caused by GLP is related to the combination of other medications, such as the combination of anticoagulant drugs [9, 43]. This bleeding may also be related to the presence of ginkgolide B, but its specific content in *Ginkgo biloba* is unknown and remains to be studied. Therefore, it may be prudent not to use GLP in combination with anticoagulants such as aspirin and warfarin and to control the dosage strictly within a reasonable range [44].

### 4.1. Research Limitations

This study provides a reference for clinical practice but also has some limitations. First, the quality of the included articles was not a consideration, the number of articles was small, and the overall sample size was also small. Second, of the 13 included articles, some may have used the wrong randomization method, while others did not. Some of them used a random number method, but none of the articles mentioned the implementation of a blind method. Third, all the included experiments were not registered for clinical trials, which could affect the study results to a certain extent, and most of the included experiments lacked safety evaluation schemes. Finally, different medications and courses of treatment in basic treatment could have led to bias in results, which can affect the reliability of the conclusions from our MA.

## 5. Conclusions

This review strengthens the evidence that GLP has a good therapeutic effect on patients with ischemic stroke. There are some limitations in our current study, but clinical trials are expected to improve the level of evidence even more through more rigorous experimental design, more comprehensive indicators, and large-sample and high-quality RCTs.

## Figures and Tables

**Figure 1:** Flow diagram of the literature screening process and results.

**Figure 2:** Risk of bias assessment for the 13 included studies.

**Figure 3:** Forest plot of NIHSS analysis.

**Figure 4:** Forest diagram of clinical therapeutic effect.

**Figure 5:** Forest plot of BI analysis.

**Figure 6:** Forest plot of plasma viscosity.

**Figure 7:** Forest plot of fibrinogen.

**Figure 8:** Forest plot of adverse reaction analysis.

**Table 1:** Details from trials.

First author, year	Reference no.	Intervention		Sample size		Age		Duration	Outcome
		Treatment	Control	Treatment	Control	Treatment	Control		
Sun T, 2012	[14]	Aspirin + ozagrel + Ginkgo dameer	Aspirin + ozagrel	40	40	66.5	64.8	2 weeks	a, b
Zhou YF, 2016	[15]	Routine + shuxuening	Routine	63	63	68.3 ± 8.5	67.1 ± 7.9	2 weeks	a, b, c
Shi YF, 2017	[16]	Routine + aspirin + ginkgo ester dispersive tablets	Routine + aspirin	41	41	69.42 ± 7.24	68.72 ± 8.14	2 weeks	d, e
Wang LM, 2017	[17]	Edaravone + propranolol + aspirin + mannitol + furosemide + *Ginkgo biloba* leaf extract	Edaravone + propranolol + aspirin + mannitol + furosemide	73	73	59.48 ± 13.24	58.91 ± 13.07	4 weeks	d, f
Yang T, 2017	[18]	Routine + alprostadil + ginkgo ester dispersive tablets	Routine + alprostadil	49	49	68.9 + 1.7	68.2 ± 1.6	2 weeks	d, f
Zhou G, 2018	[19]	Routine + rosiglitazone + ginkgo ester dispersive tablets	Routine + rosiglitazone	51	51	53.64 ± 10.25	53.72 ± 10.38	4 weeks	a, b, d, e
Zhou QW, 2019	[20]	Rt-PA + ginkgolide injection	Rt-PA	44	43	63.08 ± 7.18	62.97 ± 7.25	2 weeks	a, b
Chen E, 2020	[21]	Mannitol + aspirin + mecobalamin + ginkgo ester dropping pills	Mannitol + aspirin + mecobalamin	50	50	53.10 ± 10.39	52.39 ± 10.23	2 weeks	d, e
Xiao H, 2020	[22]	Butylphthalide + ginkgo diterpene lactone glutamine	Butylphthalide	41	41	62.15 ± 6.45	61.37 ± 6.44	2 weeks	a, b
Wu Y, 2020	[23]	Routine + ginkgolide injection	Routine treatment	46	46	68.9 + 1.7	68.2 ± 1.6	2 weeks	d, f
Zhang DN, 2020	[24]	Routine + butylphthalide + ginkgolide injection	Routine + butylphthalide	39	39	61.98 ± 7.65	61.82 ± 7.51	4 weeks	a, b, c, f
Shi XJ, 2021	[25]	Routine + Butylphthalide injection + diterpene lactone *Ginkgo biloba* injection	Routine + Butylphthalide injection	63	63	65.13 ± 7.29	64.23 ± 6.18	2 weeks	b, c, d,
Zhang TT, 2021	[26]	Rt-PA + *Ginkgo biloba* extract injection	Rt-PA	30	30	56.28 ± 5.09	56.91 ± 5.38	1 week	a, b, c, e, f

Outcomes: (a) NIHSS; (b) clinical therapeutic effect; (c) BI; (d) plasma viscosity; (e) fibrinogen; (f) adverse reactions.

## Data Availability

The datasets generated and analyzed during the current study are available in the 5 databases (details are provided in the Study Selection section).

## Abbreviations

GLP: *Ginkgo biloba* leaf preparation
RCTs: Randomized controlled trials
CNKI: China National Knowledge Infrastructure
CQVIP: Chongqing VIP
CBM: Chinese Biomedical Literature
MAs: Meta-analysis
NIHSS: National Institute of Health Stroke Scale
BI: Barthel Index.
FIB: Fibrinogen (FIB).

## References

[1] The Writing Committee of the Report on Cardiovascular Health Diseases in China (2020). Report on cardiovascular health and diseases in China 2019: an updated summary. *Chinese Circulation Journal*.

[2] Xu J., Tan S. (2016). Current status of compliance with secondary prophylactic medication in patients with ischemic stroke and transient ischemic attack. *The Journal of Practical Medicine*.

[3] Mukundan G., Seidenwurm D. J. (2018). Economic and societal aspects of stroke management. *Neuroimaging Clinics of North America*.

[4] Gong C., Hoff J. T., Keep R. F. (2000). Acute inflammatory reaction following experimental intracerebral hemorrhage in rat. *Brain Research*.

[5] He W., Wang Q. R., Zeng X. F., Lu H. (2006). Experimental research progress of treating cerebral edema after intracerebral hemorrhage with drugs for activating blood circulation and removing blood stasis. *Chinese Journal of Thrombosis and Hemostasis*.

[6] Zi Y., Liu H. F., Li Z. (2014). Effect of ginkgo biloba extract injection on hemodynamics in patients with ischemic stroke. *Journal of Clinical Rehabilitative Tissue Engineering Research*.

[7] Wang G., Yao M. J., Xu L., Cao S., Li X. F., Liu J. X. (2021). Research progress on pharmacological mechanisms of ginkgolides in the treatment of ischemic stroke. *Pharmacology and Clinics of Chinese Materia Medica*.

[8] Zheng W. R., Han Z. Z., Wang Z. K. (2019). Research advance in the safety of ginkgo biloba preparation. *Modernization of Traditional Chinese Medicine and Materia Medica-World Science and Technology*.

[9] Wang S. N. (2015). Pharmacological action and adverse reaction analysis of ginkgo biloba leaf preparation. *World Latest Medicine Information*.

[10] Koch E., Jaggy H., Chatterjee S. S. (2000). Evidence for immunotoxic effects of crude ginkgo biloba L. Leaf extracts using the popliteal lymph node assay in the mouse. *International Journal of Immunopharmacology*.

[11] Oberpichler H., Sauer D., Rossberg C., Mennel H. D., Krieglstein J. (1990). Paf antagonist ginkgolide B reduces postischemic neuronal damage in rat brain Hippocampus. *Journal of Cerebral Blood Flow and Metabolism: Official Journal of the International Society of Cerebral Blood Flow and Metabolism*.

[12] Higgins J., Green S. (2011). *Cochrane Handbook for Systematic Reviews for Interventions*.

[13] Moher D., Liberati A., Tetzlaff J., Altman D. G. (2009). Research methods and reporting. preferred reporting items for systematic reviews and meta-analyses: the prisma statement. *PLoS Medicine*.

[14] Sun T. (2012). Clinical observation of ozagrel sodium combined with ginkgo damol in the treatment of acute ischemic stroke. *China Practical Medicine*.

[15] Zhou Y. F. (2016). Effect of Ginkgo biloba extract in adjuvant treatment of senile ischemic stroke. *Chinese Journal of Rural Medicine and Pharmacy*.

[16] Shi Y. F. (2017). Effects of Ginkgo biloba dispersible tablets combined with aspirin on Hemorheology and neurological deficits in patients with ischemic stroke. *Ningxia Medical Journal*.

[17] Wang L. M., Wang Q. H. (2017). Effect of Ginkgo biloba extract on ischemic stroke and its influence on serum superoxide dismutase and malondialdehyde. *Chinese Journal of Biochemical and Pharmaceuticals*.

[18] Yang T., Yin X. X., Zhao H. (2017). Clinical study of ginkgo ester dispersive tablet combined with alprostol injection in the treatment of ischemic stroke. *Shanxi Medical Journal*.

[19] Zhou G., Li Q. (2018). Therapeutic effect of Ginkgo ketoester dispersible tablet combined rosiglitazone on patients with ischemic stroke and its influence on neurological function. *Chinese Journal of Cardiovascular Rehabilitation Medicine*.

[20] Zhou Q. W., Wang J., Wang Z. H. (2019). Clinical study of ginkgolide injection combined with alteplase intravenous thrombolysis in patients with acute ischemic stroke. *Chinese Youjiang Medical Journal*.

[21] Chen E., Liu L. P. (2020). Effect of ginkgo ester dropping pills on hemorheology and neurological function in patients with ischemic stroke. *The Medical Forum*.

[22] Xiao H., Sun N., Chen Y. Y. (2020). Clinical study of ginkgolides sodium chloride injection combined with butylphthalide in the treatment of acute progressive stroke. *Evaluation and Analysis of Drug-Use in Hospitals of China*.

[23] Wu Y., Wu Y. L., Wang S. K. (2020). Clinical effects of ginkgolide injection as an adjuvant therapy on cerebral arterial thrombosis in the elderly and its effects on neurological function and prognosis of patients. *Hebei Medical Journal*.

[24] Zhang D. N., Tian H. (2020). Clinical effect of butylphthalide soft capsule combined with ginkgolide injection in the treatment of convalescent patients with ischemic stroke. *Clinical Research and Practice*.

[25] Shi X. J., Li X. M., Yang W. J. (2021). Effect of butylphthalide injection combined with Ginkgo diterpene lactone injection on patients with acute cerebral infarction and improvement of collateral circulation. *Hebei Medical Journal*.

[26] Zhang T. T., Xi C. H., Dong B., Song D. H., Zhang L. L. (2021). Effect of ginkgo biloba extract injection combined with alteplase intravenous thrombolytic therapy on acute cerebral infarction and its effect on hemorheology and inflammatory factors. *Progress in Modern Biomedicine*.

[27] Xu J. H., Xu Y. H., Cai Z. R., Yu M. (2019). Comparison of efficacy and safety of three different antithrombotic drugs for secondary prevention of ischemic stroke in patients with NVAF. *Jilin Medical Journal*.

[28] Zhang Y. B. (2019). Effect of intravenous thrombolysis of ligustrazine hydrochloride combined with alteplase in patients with acute ischemic stroke. *Henan Medical Research*.

[29] Zhu J., Guo S., Zhao L., Zhu Y. B. (2020). Efficacy of intensive medical treatment regimen in the acute phase of ischemic stroke. *Journal of Chengdu Medical College*.

[30] Tran H., Anand S. S. (2004). Oral antiplatelet therapy in cerebrovascular disease, coronary artery disease, and peripheral arterial disease. *Journal of the American Medical Association*.

[31] Friend M., Vucenik I., Miller M. (2003). Research pointers: platelet responsiveness to aspirin in patients with hyperlipidaemia. *BMJ (Clinical research ed.)*.

[32] Cambria-Kiely J. A., Gandhi P. J. (2002). Possible mechanisms of aspirin resistance. *Journal of Thrombosis and Thrombolysis*.

[33] Liu Q. K., Wang Z., Xie J., Liu M., Zou W. H. (2010). A controlled clinical study of ginkgo biloba leaf in the treatment of aspirin resistance. *Zhejiang Journal of Traditional Chinese Medicine*.

[34] Yang H. J., Huang H. P., Xu H. F. (2011). Aspirin combined with ginkgo biloba preparation reduced aspirin resistance in 50 cases. *Herald of Medicine*.

[35] Liu X. P., Zang H. C., Yu H. L. (2014). Research progress and application prospect of ginkgo biloba leaf extract. *Journal of Pharmaceutical Research*.

[36] Zhuo B., Mei Q. X. (2001). Pharmacology and clinical study of ginkgo biloba leaf extract. *China Pharmaceuticals*.

[37] Xu L., Hu Z., Shen J., McQuillan P. M. (2015). Effects of ginkgo biloba extract on cerebral oxygen and glucose metabolism in elderly patients with pre-existing cerebral ischemia. *Complementary Therapies in Medicine*.

[38] Liu GL. (2016). Pharmacological action and clinical application of Ginkgo biloba preparation. *Shanghai Medical & Pharmaceutical Journal*.

[39] Hu T. (2020). Changes and value of serum CRP, D-dimer, lipoprotein A and fibrinogen in patients with ischemic stroke. *Chinese Journal of Public Health Engineering*.

[40] Zhang F. J., Li X. M., Zhang J., Wang A. M., Zhou L. P., Li X. G. (2019). Levels of D-dimer, fibrinogen, and fibrinogen degradation product in patients with acute chest pain. *Journal of Central South University*.

[41] Zhang SY. (2019). Advances in pharmacological and toxicological effects and deacidification methods of ginkgolic acids. *Chinese Community Doctors*.

[42] Zhang X. F., Hu J. T., Jia S. K., Lin Y. R., Ouyang J. F. (2020). Commentary on the pharmacology, efficacy, toxicity and edible safety of. *Forum on Traditional Chinese Medicine*.

[43] Wei L. H., Li Y. (2007). Pharmacological effects and adverse reactions of ginkgo biloba leaf preparation. *Strait Pharmaceutical Journal*.

[44] Chinese Medical Association Branch of Integrated Traditional Chinese and Western Medicine (2020). Chinese experts consensus on clinical application of oral ginkgo biloba preparations. *Chinese Journal of Integrated Traditional and Western Medicine*.

